# Artificial Intelligence-Based Echocardiographic Left Atrial Volume Measurement with Pulmonary Vein Comparison

**DOI:** 10.1155/2021/1336762

**Published:** 2021-12-06

**Authors:** Mengyun Zhu, Ximin Fan, Weijing Liu, Jianying Shen, Wei Chen, Yawei Xu, Xuejing Yu

**Affiliations:** Department of Cardiology, Shanghai Tenth People's Hospital, Tongji University School of Medicine, Shanghai 200072, China

## Abstract

This paper combines echocardiographic signal processing and artificial intelligence technology to propose a deep neural network model adapted to echocardiographic signals to achieve left atrial volume measurement and automatic assessment of pulmonary veins efficiently and quickly. Based on the echocardiographic signal generation mechanism and detection method, an experimental scheme for the echocardiographic signal acquisition was designed. The echocardiographic signal data of healthy subjects were measured in four different experimental states, and a database of left atrial volume measurements and pulmonary veins was constructed. Combining the correspondence between ECG signals and echocardiographic signals in the time domain, a series of preprocessing such as denoising, feature point localization, and segmentation of the cardiac cycle was realized by wavelet transform and threshold method to complete the data collection. This paper proposes a comparative model based on artificial intelligence, adapts to the characteristics of one-dimensional time-series echocardiographic signals, automatically extracts the deep features of echocardiographic signals, effectively reduces the subjective influence of manual feature selection, and realizes the automatic classification and evaluation of human left atrial volume measurement and pulmonary veins under different states. The experimental results show that the proposed BP neural network model has good adaptability and classification performance in the tasks of LV volume measurement and pulmonary vein automatic classification evaluation and achieves an average test accuracy of over 96.58%. The average root-mean-square error percentage of signal compression is only 0.65% by extracting the coding features of the original echocardiographic signal through the convolutional autoencoder, which completes the signal compression with low loss. Comparing the training time and classification accuracy of the LSTM network with the original signal and encoded features, the experimental results show that the AI model can greatly reduce the model training time cost and achieve an average accuracy of 97.97% in the test set and increase the real-time performance of the left atrial volume measurement and pulmonary vein evaluation as well as the security of the data transmission process, which is very important for the comparison of left atrial volume measurement and pulmonary vein. It is of great practical importance to compare left atrial volume measurements with pulmonary veins.

## 1. Introduction

In recent years, the procedure has been gradually refined and matured and has demonstrated more outstanding safety and efficacy than traditional drug therapy, leaping to become the first-line treatment option for patients with atrial fibrillation [1]. The increase in the surgical base has also led to a relative increase in complications, which include pulmonary vein stenosis (PVS), pericardial effusion, arteriovenous embolism, and atrioventricular oesophageal fistula. The cardiac impedance signal is an impedance change signal measured directly from the body surface of the human chest using bioimpedance technology. Since the cardiac impedance signal has no negative waveform, it is often differentiated to reflect the pumping function of the heart from a hemodynamic perspective [2]. The pumping function of the heart can effectively reflect the location of the lesion in patients with cardiovascular diseases, the physical condition of the body, and the level of exercise training and is one of the important reference bases for the diagnosis of various cardiovascular diseases [3, 4]. Therefore, left atrial volume measurement and pulmonary vein assessment are of great importance for guiding treatment and assessing the functional status of the heart in patients with cardiovascular diseases. Artificial neural networks propose the concept of deep learning, which intends to make the machine simulate the multilayered information processing of the brain and automatically extract the intrinsic laws and representation levels of the input data through training [5]. With the rapid development of deep neural networks, their applications in the medical field are becoming more and more widespread, with relevant applications in disease diagnosis, medical image segmentation, drug tracking, medical text analysis, clinical aid diagnosis, treatment, and so forth. The launch of the AI intelligent imaging platform has brought new research ideas in human medical health assessment intelligence.

Some machine learning techniques help determine the sources and sequence variables that play an important role in the cause of the disease. In supervised learning, the algorithm consists of input and output, and the goal is to map input to output. It has a wide range of clinical applications, such as image recognition, interpretation of patients' electrocardiograms, chest X-rays, and CT results. In supervised learning, a set of databases containing observation data and their results can be used to build a predictive model that can classify the results from another set of given observation data [6]. The goal of unsupervised learning is to understand the internal relationships and patterns of the data itself. However, there is a lack of quantitative measurements of the relationship between parameters and prognostic status and a lack of comprehensive evaluation of the comparative ability of each parameter. Therefore, the development of a prognostic model for heart failure patients based on echocardiographic metrics is of great value to assist clinicians in the treatment of hospitalized patients and the daily management of patients after discharge. Comparative models were developed by applying machine learning algorithms with traditional statistical methods, that is, logistic linear regression, respectively, and, by comparing the values of the two models developed for the assessment of mortality and the risk of cardiovascular events in patients, it was concluded that comparative risk models with good comparative power and risk identification could be obtained by machine learning algorithms [7]. The purpose of this paper is to establish a comparative model based on the echocardiographic findings of the patients, by applying the BP neural network learning algorithm jointly by applying the 7 indicators reflecting the cardiac function of the patients obtained by echocardiography, and to conduct a comparative study on the comparative results of patients with reduced ejection fraction, that is, 1-year readmission and 3-year mortality, which has high clinical research and practical application significance.

The echocardiographic technique, as a clinical medical test for a comprehensive understanding of cardiac structure and function, has not been effectively used in left atrial volume measurement and pulmonary vein comparison. This study uses the echocardiographic technique for comprehensive observation of cardiac morphology and function, making the means of left atrial volume measurement and pulmonary vein comparison more accurate, efficient, and novel. Cardiac echocardiography is widely used in clinical medicine as the optimal test for determining the morphology and function of the heart. The first chapter firstly discusses the background and research significance of cardiovascular diseases, clarifies the main problems at the present stage, and clarifies the research plan and the chapter arrangement of the whole paper. The second chapter provides a brief review of the current state of development of domestic and international research on artificial intelligence for echocardiography, left atrial volume measurement and pulmonary vein assessment and detection methods, and deep learning. The third chapter proposes a 1D-CNN comparison model from deep neural networks, combining the characteristics of cardiac impedance differential signals themselves, to automatically learn the waveform features of cardiac impedance differential signals and avoid the manual feature selection process. Firstly, the cardiac impedance database is preprocessed, including signal denoising, feature point localization, and signal segmentation, to complete the data preparation work. The fourth chapter evaluates the model performance by test set samples and provides a detailed description and analysis of the experimental results. Then, the left atrial volume measurement and pulmonary vein classification in different states of the human body are evaluated by deeply mining the temporal connections between data points through long short-term memory networks. Finally, the validity of the model is verified by comparing the original data with the signal encoding features. The fifth chapter summarizes the research content of this paper.

## 2. Related Work

Echocardiography (UGG) is a noninvasive test that uses ultrasound echoes to examine the heart and large blood vessels to obtain relevant information. The echocardiogram provides information not only on the morphology and structure of the heart but also on the function of the heart and is an effective tool for evaluating the functional status of the heart. Quer et al. used X-ray fluoroscopy to find a strong heartbeat in humans and confirmed cardiac hypertrophy using X-ray until the introduction of echocardiography, which was a major step forward in the study of the heart [8]. Lai W T et al. began examining the heart using M-mode echocardiography and found that left ventricular hypertrophy was more common in humans in strength training programs [9]. Liu et al. further confirmed the enlargement of the heart ventricles in endurance training programs using two-dimensional echocardiography. Echocardiography not only allows for the evaluation of cardiac morphology and function but also allows for the accurate identification of cardiac and pathological hearts, which can effectively prevent the occurrence of sudden cardiac death in humans while guiding them through exercise training [10]. Cardiac enlargement and myocardial hypertrophy have been shown to occur in humans with prolonged exercise training, and the hypertrophy is often accompanied by an abnormal electrocardiogram, similar to that seen in clinical hypertrophic cardiomyopathy [11, 12].

Neural networks have been widely used in cardiovascular disease to quantify the complex relationships between the given data and have shown superior comparative ability in many areas such as diagnosis, response to treatment, and prognosis for patients suffering from various diseases [13]. Gearhart et al. used neural networks and cardiopulmonary function tests to compare the risk of cardiovascular-related mortality in patients who had heart failure with a left cardiopulmonary function test were followed up, and the results of the obtained tests and patient survival were composed into a sample set, which was randomly divided into a training set and a test set to compare cardiovascular-related mortality [14]. Olier et al. applied a cardiac hemodynamic monitor to measure left atrial volume measurements and pulmonary vein parameters by the cardiac impedance method in patients with coronary artery disease at different times to observe the effects of coronary artery disease on patients' left atrial volume measurements and pulmonary veins to further guide clinical diagnosis [15]. Chaturvedi et al. measured the hemodynamic indexes of heart failure patients by impedance hemogram detector and correlated them with BNP and left ventricular ejection fraction to explore their clinical significance in left atrial volume measurement and pulmonary vein assessment. Li et al. proposed BiLSTM-Attention neural network model with the heartbeat to improve the classification accuracy of heartbeat ECG signal [16]. La Porta E et al. used a 34-layer deep convolutional neural network trained on a dataset of 9123 ECG recordings from approximately 40,000 patients to achieve the classification of 15 rhythm types. From the above studies, it can be seen that, with the continuous development of deep learning, the use of deep learning methods in the medical field to mine the deep information of medical data and assist doctors in diagnosis and treatment has become a hot spot at home and abroad [17].

This paper adopts deep learning method to study and analyze the left atrial volume measurement and pulmonary vein status of the human body under the different intensity of exercise based on cardiac impedance differential signal and design a completely automatic feature learning model of cardiac impedance differential signal to reflect the effect of different intensity on the dynamic changes of cardiac blood flow and complete the automatic classification assessment of left atrial volume measurement and pulmonary vein function, which has the functions of real-time monitoring, predisease warning, and medical aid diagnosis [18, 19]. The db6 wavelet transform was used to decompose the signals in 8 layers, remove the signal noise at different frequencies, locate the signal characteristics and segment the signals, and establish the cardiac impedance database. The cross-validation method is used to divide 85% of the data samples into training and validation sets to test the model training, and the remaining 15% of the data samples are used as a separate test set to test the model generalization ability, evaluate the model performance, and complete the data preparation work [20, 21]. Finally, the deep left atrial volume measurement and automatic pulmonary vein assessment models are designed based on deep learning methods combined with one-dimensional cardiac impedance differential signal features [22]. According to the current experimental conditions, the use of cardiac echocardiography to compare the left atrium volume measurement with the pulmonary vein will provide experimental support and practical guidance for scientific exercise training monitoring and exercise plan formulation.

## 3. Artificial Intelligence-Based Echocardiographic Left Atrial Volume Measurement and Pulmonary Vein Comparison Study

### 3.1. Artificial Intelligence-Based Echocardiographic Parameter Building

After confirming that the electrodes and interfaces are correctly connected, the AcqKnowledge physiological signal acquisition software is used to synchronize the signal acquisition, convert the cardiac impedance signal and ECG signal into digital signals at the same time, and create a new channel to differentiate the cardiac impedance signal to obtain the cardiac impedance differential signal waveform. As shown in Figure 1, channel 2 is the cardiac impedance signal waveform, channel 10 is the cardiac impedance differential signal waveform, and channel 11 is the electrocardiographic signal waveform.

BP neural networks need to be trained before they can be used in comparison studies, to obtain networks with the ability to make accurate comparisons as well as associations with unknown data [23]. M is set as the input data and N is set as the output data, and the number of nodes in each layer is set as *x*, *l*, and *y* according to the provided sample data, after which the appropriate weights *w*_*ij*_ and *w*_*jk*_ between the layers are set according to the situation, and the thresholds *x* and *y* for the implicit and output layers are set, after which the learning rate and the relatively appropriate neuron excitation functions are selected according to the set target requirements.

The output *Z* of the intermediate hidden layer is obtained by basing on the input data M the threshold *m* of the next layer and *w*_*ij*_ between the two layers, as shown in the following equation:

(1) $$\begin{array}{c} Z_{j}=g\left(\sum_{i=1}^{n}w_{ij}*m_{i}-x_{j}\right)\;j\subseteq \left[1,l\right]. \end{array}$$

In equation (1), *m* is the excitation function of the implicit layer in the middle, multiple functions can be selected to execute. According to the research purpose of this paper, our definition is as follows:

(2) $$\begin{array}{c} \cos\left(m\right)=\frac{3-\alpha *x}{1+\exp\left(-3x\right)\left(mx-nx\right)}. \end{array}$$

Based on *Z* obtained above, threshold *y* of the next layer, and *w*_*jk*_ between the two layers, the comparison result of this network is obtained after processing *P*(*k*).

(3) $$\begin{array}{c} P\left(k\right)=\sum_{j=1}^{l}\left(Z_{j}*w_{jk}-n_{k}\right),\;k\subseteq \left[1,m\right]. \end{array}$$

The new processed weights *w*_*ij*_ and *w*_*jk*_ are obtained by the error as in equation (4), and *n* is the set learning rate.

(4) $$\begin{array}{c} \left\{\begin{array}{c} w_{ij}=\psi *Z_{j}\left(1-Z_{j}\right)*\sum_{j=1}^{n}w_{ij}*e_{j},\\ w_{jk}=\psi *Z_{j}*e_{k}. \end{array}\right) \end{array}$$

The errors are used to obtain the new threshold values *x* and *y* after processing, as in equation (5). Determine the current iteration of the algorithm to reach the target, the algorithm iterations, that is, the old values, are used to continuously recursively get new values, and the purpose of this process is to confirm whether the desired output can be reached. If the target is not reached, it returns to continue the training.

(5) $$\begin{array}{c} \left\{\begin{array}{c} x_{j}=\psi *Z_{j}\left(1-Z_{j}\right)*\sum_{j=1}^{n}w_{ij}*e_{j}+m_{j},\\ y_{k}=n_{k}+e_{k}. \end{array}\right) \end{array}$$

Input parameters were selected for this study based on 7 relevant indices obtained by echocardiography: left ventricular end-diastolic internal diameter size, left ventricular ejection fraction size, pulmonary artery systolic pressure size, mitral regurgitation degree grouping, and tricuspid regurgitation degree grouping, with or without pericardial effusion and with or without pleural effusion confirmed by combined chest radiographs [24, 25]. *Q* (the number of neurons in the hidden layer) was determined based on equation (6). *X* and *Y* were the number of indicators of the input echocardiogram and the prognosis of the set heart failure patients, respectively.

(6) $$\begin{array}{c} Q=\max\left(X\left(Y+1\right),2X,Y\left(X+1\right),3Y\right). \end{array}$$

Because of the large gap between the data of each echocardiographic index and the values of 1-year readmission and survival time as the results, the accuracy of the comparison results of heart failure patients may be affected during the network processing, so all the echocardiographic indexes and the prognostic results of patients should be normalized uniformly, and the data information of all patients should be transformed into a number between [0, 1], and the maximum-minimum method is applied here; min(B) is the smallest value among all data of each echocardiographic index, and max(B) is the largest value among all results of each prognostic condition, and the data obtained after the transformation can be directly used for the training of the following neural network:

(7) $$\begin{array}{c} AI=\frac{\left(B-\min\left(B\right)\right)}{\left(\max\left(B\right)\left(\right)-\min\left(B\right)\right)}. \end{array}$$

After the weights and thresholds obtained through multiple trainings meet the identified target requirements, they are used as the parameters of the prognostic prediction model and placed in the network. It can better perform echocardiographic left atrial volume measurement and comparison with pulmonary veins. The next step is to set the training parameters of this heart failure prognostic comparison model: step size and learning rate. The learning rate should be set to a small value because a larger value will speed up the convergence at the beginning of the training, but it will not converge when it is close to the optimal value. Automatically extract the internal laws and representation levels of the input data through training.

### 3.2. Left Atrial Volume Measurement and Pulmonary Vein Comparison Method

After the subjects were identified through the questionnaire, the test time was determined through communication with the subjects to ensure that the subjects did not perform any training the day before, and the experimental group was allowed to sit still for at least 5 minutes before the test. A physician was in front of the computer and color printer to enter the information, record the data, and print the color echocardiography report form of the Hospital, and the control group was tested in the same way as the experimental group.

The left ventricular long-axis view measured the left atrial anterior-posterior diameter (LAAPD), left ventricular end-diastolic internal diameter (LVEDD), and left ventricular end-systolic internal diameter (LVESD); the apical four-chamber view measured the left atrial left-right diameter (LALRD) and left atrial upper and lower diameters (LASID); the real-time biplane method measured the left atrial maximum volume (LAVmax) at end-systole and the left atrial minimum volume (LAVmin) at end-diastole. LAVmax was measured at end-systole, LAVmin was measured at end-diastole, and LAVp was measured at the beginning of the P wave of the electrocardiogram, which could not be measured in PeAF patients without preoperative P wave. The shape of the pulmonary vein inlet is observed and measured by adjusting it at different angles. The disadvantage is that only one profile of the vessel can be displayed, so the accuracy of the operation affects the accuracy of the measurement results.

In pulmonary vein and left atrium imaging, the anatomical structure of the pulmonary vein vestibule can be directly observed by VE technique (comprehensive use of computer graphics systems and various reality and control interface devices to provide immersive technology in an interactive three-dimensional environment generated on a computer; among them, the computer-generated, interactive three-dimensional environment becomes a virtual environment), and the morphology and location of the intrapulmonary vein crest can be visualized, and the number of pulmonary vein openings can be clarified; it is also possible to clarify whether a small variant vein, which cannot be accurately displayed in postprocessing techniques such as VR and MPR, or a branch adjacent to the root of the pulmonary vein, is a variant by observing the location of the internal entrance of the vessel. The position of the interventricular ridge can also be used as an observation marker to further clarify whether the vein is a common pulmonary vein, which should project into the lumen of the left atrium if it is not a common pulmonary vein or deeper into the lumen of the pulmonary vein if it is a common pulmonary vein. The flow of left atrial volume measurements compared with pulmonary veins is shown in Figure 2. In patients with atrial electrical remodeling and an enlarged pulmonary vein inlet, atrial fibrillation cannot be completely cured by pulmonary vein isolation alone with atrial fibrillation ablation because of the presence of ectopic potential trigger points; and the enlarged pulmonary vein inlet may also affect the increase in electrical remodeling. The enlargement of the pulmonary vein inlet may lead to the easier formation of residual electrical conduction between the ipsilateral pulmonary veins and more likely to lead to ectopic trigger points outside the pulmonary veins. The increased diameter of the pulmonary vein entrance lengthens the ablation path; it becomes more difficult to keep all ablation points in the same plane during intraoperative ablation, resulting in a decreased success rate. The enlargement of the pulmonary vein entrance increases the number of atrial fibrillation trigger points and electrical activity, thus increasing the difficulty and complexity of the procedure and decreasing the success rate of the procedure.

A combination of postprocessing techniques and a comprehensive analysis is required for more objective and accurate observation and measurement of the pulmonary veins. When measuring the pulmonary vein inlet diameter in the transverse axis of the original image, it is difficult to observe the exact location of the opening because some of the left atrial walls are gently displaced from the pulmonary veins, and the presence of the left ventricle also makes it difficult to measure the left upper pulmonary vein. When measuring the pulmonary vein inlet diameter on VR images, although it can be rotated in multiple angles, it is difficult to select the starting and ending points for the measurement because it is modeled in three dimensions. When measuring the pulmonary vein inlet diameter on MIP images, care should be taken to avoid overlapping vascular images around the measurement results because of the density of the image. When measuring the pulmonary vein inlet diameter on MPR images, the division between the pulmonary vein inlet and the left atrium can be clearly shown, but because it is a two-dimensional reconstruction image, there is some image distortion on the image, which may affect the measurement results. When measuring the pulmonary vein inlet diameter on VE images, the structures within the pulmonary vein lumen can be seen, but because it is a real-time speculum image, care should be taken to determine the edge of the pulmonary vein inlet by rotating it at different angles.

In this study, both direct and indirect contrast methods were used to measure the narrowed pulmonary veins. The direct contrast method is the most classic method of PVS measurement, which has the advantage that preoperative and postoperative data can be retrieved and analyzed simultaneously to exclude the presence of preoperative PVS and pulmonary vein malformation; the disadvantage is that if the difference between the two imaging methods is large, the measurement results will be different, which will affect the PVS staging and the next treatment plan. The advantage of the indirect contrast method is that the presence of PVS can be inferred from postoperative CTA alone and the degree of stenosis can be calculated without obtaining additional preoperative data, which is suitable for patients with missing preoperative imaging data or with large differences between preoperative and postoperative imaging data. However, this method cannot exclude the existence of preoperative PVS and pulmonary vein malformation, and the conclusion is relatively one-sided. However, combined with the actual clinical situation, many patients were unable to provide preoperative imaging data at the time of follow-up due to the different locations of surgery and follow-up. Therefore, this study used both measurement methods to assess the degree of pulmonary vein stenosis and compared the two methods, aiming to demonstrate that, for patients who underwent CPVI for the first time, the occurrence of PVS can also be determined using only the indirect comparison method. However, the presence of special cases should also be considered in the clinical application, if the patient has missing preoperative data and develops postoperative chest tightness, cough, dyspnea, palpitations, difficult to specify etiology of recurrent pulmonary infections, and other symptoms; even if no obvious PVS is seen by indirect comparison method, the presence of PVS should be considered for further examination and follow-up.

## 4. Results and Analysis

### 4.1. Analysis of Simulation Results

First, the heart rate and the basic parameters of BSA and BV were calculated for each subject in the natural lying breathing state, as shown in Figure 3. The first 6 of the 20 subjects shown in Figure 3 were 12 female and the last 8 subjects were male. The mean heart rate of the female subjects was 76.74 beats/min and the mean heart rate of the male subjects was 74.12 beats/min, which were within the normal range of heart rate in the natural quiet state. In addition, because the heart volume of female subjects was slightly smaller than that of male subjects, the pumping capacity of the myocardium was relatively weaker, and the heart of female subjects needed to pump more times at the same time to ensure normal blood supply. Therefore, the average heart rate of female subjects was slightly faster than that of male subjects, and all measured data were within the normal heart rate reference range.

To further evaluate the effectiveness of convolutional self-coding structure as a signal compression method and signal coding features, and to facilitate the comparison and analysis of experimental results, two LSTM classification network models are prepared in this paper for comparison and evaluation. The only difference between the two networks is that the input signals are different. In the training phase of the model, the same tenfold cross-validation method is used to divide the training and validation sets for 85.14% of the data samples, and the remaining 15.14% are used for testing. Using the Adam optimizer, the batch size is 50.2; models are trained for 2000 iterations and the classification performance of the training model is evaluated using the test data, and the training results of the 2 models are presented in Figure 4.

The model test accuracy further verifies that the convolutional self-coding extracts effective coding features of the cardiac impedance differential signal. In terms of model training time, the former model takes 8635.12 seconds or 2.40 hours to achieve 10,000 iterations, while the latter only takes 1328.27 seconds or 0.37 hours, which is about 6.5 times longer than the latter. The greatly reduced model training time indicates that the CLSTM model can minimize storage requirements, reduce data transfer costs and hardware configuration requirements, and improve real-time performance. In addition, the data is transmitted in encoded form to enhance data security. The evaluation parameters corresponding to each category are calculated based on the confusion matrix, as shown in Figure 5.

The model automatically learns the deep-level encoding features of the cardiac impedance differential signal through the convolutional autoencoder, which effectively compresses the cardiac impedance differential signal, reduces the model computational complexity, and decreases the model training time. Through a feedback mechanism, a 5-layer LSTM is used to integrate the valuable memories stored in the past and the contextual state of the current moment to deeply explore the strong correlation between the data points of the cardiac impedance differential signal and complete the classification assessment of cardiac function in different states of the human body. The average accuracy of the test set is 98.18% and 97.87%, and the training time of the model is reduced from 2.4 hours to 0.37 hours, indicating that the CLSTM model proposed in this paper has stronger real-time performance and lower hardware requirements.

### 4.2. Analysis of Comparative Results

For maximum diameter of pulmonary vein openings in the paroxysmal and continuous groups, LSPV was the largest, followed by RSPV, and LIPV and RIPV were the smallest; for the minimum diameter of pulmonary vein openings, RSPV and RIPV were the largest, followed by LSPV, and LIPV was the smallest; for the mean diameter, circumference, and area of pulmonary vein openings, RSPV and LSPV were the largest, followed by RIPV, and LIPV was the smallest; There were statistical differences in pulmonary vein openings (*P* < 0.05), as shown in Figure 6(a). In the normal control group, for the maximum diameter of pulmonary vein opening, RSPV and LSPV were the largest, followed by RIPV, and RSPV was the smallest; for the minimum diameter, mean diameter, circumference, and area of pulmonary vein opening, RSPV, RIPV, and LSPV were larger than LIPV; for the degree of incompatibility of pulmonary vein opening, LSPV and LIPV were the largest, followed by RSPV, and RIPV was the smallest; for the length of pulmonary vein trunk, LSPV and LIPV were the largest, followed by RSPV, and RIPV was the smallest. All of them were statistically different (*P* < 0.05), as shown in Figure 6(b).

For comparison of pulmonary vein opening sizes, the results of the maximum diameter, minimum diameter, mean diameter, circumference, and area of the LSPV and LIPV openings were statistically different among the three groups (*P* < 0.05), and the continuous group was larger than the normal and paroxysmal groups; the results of the above diameters of the RSPV and RIPV openings were not statistically different (*P* > 0.05). In the normal, paroxysmal, and persistent groups, the upper and lower left atrial diameters were 57.8 mm, 61.3 mm, and 62.6 mm, respectively, and there was a statistical difference between the three groups (*P* < 0.05), and the paroxysmal and persistent AF groups were larger than the normal group. The left atrial, left, and right diameters were 42.5 mm, 47.4 mm, and 43.4 mm, respectively; the anterior and posterior diameters were 32.2 mm, 36.4 mm, and 41.0 mm, respectively; and the left atrial volumes were 45.3 mm, 42.5 mm, and 48.5 mm, respectively. There was a statistical difference between the three groups (*P* < 0.05), and the sustained group was greater than the paroxysmal group and the normal group, as shown in Figure 7.

As shown in Figure 8, the cardiac echocardiographic results of female subjects in different groups showed highly significant differences (*P* < 0.01, *P* < 0.01, and *P* < 0.01) in the left ventricular septal thickness index, compared with the control group (C-F group), and in the A-F group, R-F group, and M-F group. For the left atrial anterior-posterior diameter index, the left ventricular anterior-posterior diameter was 30.3 mm in the M-F group with a highly significant difference (*P* < 0.01) compared with the control group (C-F group), and the left ventricular anterior-posterior diameter was 28.5 mm in the R-F group with a highly significant difference (*P* < 0.01) compared with the M-F group. Compared with the control group (C-F group), the left atrial, left, and right diameters in the A-F group and the R-F group were very significantly different (*P* < 0.01 and *P* < 0.01); compared with the A-F group, the R-M group, and the M-F group, they were very significantly different (*P* < 0.01 and *P* < 0.01); compared with the M-F group, the A-F group, and the R-F group, they were very significantly different (*P* < 0.01 and *P* < 0.01); compared with the M-F group, the A-F group, and the R-F group, the difference was highly significant (*P* < 0.01 and *P* < 0.01, respectively). Compared with the control group (C-F group), the upper and lower left atrial diameters were 47.4 mm in the A-F group, with a highly significant difference (*P* < 0.01), and in the R-F and M-F groups, with a highly significant difference (*P* < 0.05 and *P* < 0.05); compared with the A-F group, the R-F, and M-F groups, with a highly significant difference (*P* < 0.05, *P* < 0.01, and *P* < 0.01); compared with the A-F group, the R-F group, and the M-F group, there was a very significant difference (*P* < 0.01). For the left ventricular posterior wall thickness index, there were highly significant differences in the A-F, R-F, and M-F groups compared with the control group (C-F group) (*P* < 0.01, *P* < 0.01, and *P* < 0.01). Compared with the control group (C-F group), the left ventricular end-diastolic internal diameters of the A-F group and R-F group were significantly different (*P* < 0.05 and *P* < 0.05), and the left ventricular end-diastolic internal diameter of the M-F group was 45.6 mm, which was very significantly different (*P* < 0.01); compared with the M-F group, the left ventricular end-diastolic internal diameter of the R-F group was 43.6 mm, which was very significantly different (*P* < 0.01). The end-diastolic internal diameter of the left ventricle in the R-F group was 43.6 mm compared with that in the M-F group, with a highly significant difference (*P* < 0.01). Compared with the control group (C-F group), the left ventricular end-systolic internal diameter in the A-F group was 27.8 mm, with a significant difference (*P* < 0.05), and in the R-F and M-F groups, with a highly significant difference (*P* < 0.01 and *P* < 0.01).

Artificial intelligence technology, as a relatively new research direction, plays a role in several fields. At present, artificial intelligence technology has been widely used in the medical field and has demonstrated its value in many aspects such as diagnosis and treatment of acute or chronic diseases and prognosis evaluation. Neural network learning algorithm as one of the machine learning methods is also widely used. Neural networks are designed to analyze and process the given data by stimulating the activity of the human brain, and they have the same ability to learn by experience as that of the human brain. The echocardiographic left atrial volume measurement and pulmonary vein comparison model based on the neural network learning algorithm used in this study is suitable for dealing with the most complex nonlinear correlation problems seen in real practice, unlike the various risk comparison methods currently available, and provides a way to overcome the limitations of traditional statistical methods.

## 5. Conclusion

Echocardiographic indicators are of high value in determining the prognosis of patients, and neural network learning algorithms and other machine learning algorithms have proven their value in many fields of medicine. The MP160 multichannel physiologic meter can be used to measure the prognosis of heart failure patients. The MP160 multichannel physiological instrument was used to measure 20 subjects, and simultaneous data acquisition of cardiac impedance differential signals and ECG signals was performed. The noise interference sources contained in the collected cardiac impedance differential signals and ECG signals were analyzed, and the db6 wavelet function was selected to filter the noise within the collected data by comparing and analyzing the filtering of different wavelet bases on the collected data. The Mexican Hat wavelet transforms and the modal maximum threshold method were combined to locate the feature points of the acquired data. To further clarify the location of the feature points of the cardiac impedance differential signal, a secondary calibration of the feature points of the cardiac impedance differential signal was performed by the correspondence between the synchronized acquired ECG signal and the cardiac impedance differential signal in the time domain. The signal is segmented based on the cardiac period to increase the data sample size for the subsequent algorithm of fine identification. Finally, the data are organized and a database of cardiac impedance differential signals is established to complete the data preparation. In the future, through deep neural network and big data analysis technology, a large amount of data analysis will be carried out on the anatomy of the pulmonary veins to further clarify the relationship between the structure of the pulmonary veins and echocardiography and provide more powerful clues for medical prevention and treatment.

## Figures and Tables

**Figure 1:** Cardiac synchronized cardiac impedance signal waveform.

**Figure 2:** Left atrial volume measurements compared with pulmonary veins.

**Figure 3:** Calculated heart rate and BSA and BV parameters in the natural lying state.

**Figure 4:** Training results of LSTM classification network with different inputs.

**Figure 5:** Relevant evaluation parameters of the network test set.

**Figure 6:** Maximum diameter of pulmonary vein opening. (a) Paroxysmal group and continuous group and (b) Normal control group.

**Figure 7:** Comparison of pulmonary vein opening size and intergroup comparison of each diameter and volume of the left atrium (mm). (a) Normal group, (b) Burst group and (c) Continuous group.

**Figure 8:** Echocardiographic results of morphological indicators of the heart (mm).

## Data Availability

The data used to support the findings of this study are available from the corresponding author upon request.
